# Cystic fibrosis: current therapeutic targets and future approaches

**DOI:** 10.1186/s12967-017-1193-9

**Published:** 2017-04-27

**Authors:** Misbahuddin M. Rafeeq, Hussam Aly Sayed Murad

**Affiliations:** 1 Department of Pharmacology, Faculty of Medicine, King Abdulaziz University, Rabigh Campus, Jeddah, 21589 Saudi Arabia; 2 Department of Pharmacology, Faculty of Medicine, Ain Shams University, Cairo, 11562 Egypt

**Keywords:** Chloride, Sweat, Respiratory, Hereditary, CFTR

## Abstract

**Objectives:**

Study of currently approved drugs and exploration of future clinical development pipeline therapeutics for cystic fibrosis, and possible limitations in their use.

**Methods:**

Extensive literature search using individual and a combination of key words related to cystic fibrosis therapeutics.

**Key findings:**

Cystic fibrosis is an autosomal recessive disorder due to mutations in CFTR gene leading to abnormality of chloride channels in mucus and sweat producing cells. Respiratory system and GIT are primarily involved but eventually multiple organs are affected leading to life threatening complications. Management requires drug therapy, extensive physiotherapy and nutritional support. Previously, the focus was on symptomatic improvement and complication prevention but recently the protein rectifiers are being studied which are claimed to correct underlying structural and functional abnormalities. Some improvement is observed by the corrector drugs. Other promising approaches are gene therapy, targeting of cellular interactomes, and newer drugs for symptomatic improvement.

**Conclusions:**

The treatment has a long way to go as most of the existing therapeutics is for older children. Other limiting factors include mutation class, genetic profile, drug interactions, adverse effects, and cost. Novel approaches like gene transfer/gene editing, disease modeling and search for alternative targets are warranted.

## Introduction and pathophysiology

Cystic fibrosis (henceforth CF) is autosomal recessive disease involving mucus and sweat producing cells affecting multiple organs with lungs most severely affected leading to death in 90% of patients [1]. A mutation in Cystic fibrosis trans-membrane conductance regulator (henceforth CFTR) gene changes a protein (a regulated chloride channel), which regulate the activity of other chloride and sodium channels at the cell surface epithelium [2–4]. There are about 70,000 worldwide cases and approximately 1000 new cases are added each year. CF is most common in white people of north European ancestry having 1 in 2000–3000 births [5] and least in Asian-Americans having 1:30,000 newborns [6].

The CFTR protein lets chloride to pass through the mucus producing cells after which the water follows and mucus becomes thin. However, defective CFTR results in thick and sticky mucus obstructing the pathways [7], leading to serious lung infections especially pseudomonas. There is massive neutrophil infiltration releasing elastase, which overpowers the lung antiproteases contributing to tissue destruction [8]. Additionally, degranulating neutrophils release large quantities of nucleic acids and cytosol matrix proteins contributing to the mucus hyper-viscosity [9].

In the GIT, the mucous plugs obstruct the canaliculi of pancreas and gall bladder duct preventing enzyme and bile flow into duodenum triggering malabsorption and digestion abnormalities. Additionally, Distal Intestinal Obstruction Syndrome (DIOS), which is distinctive to CF, may occur especially in those with pancreatic insufficiency. This is characterized by ileo-cecal obstruction of inspissated intestinal contents [10, 11]. There is also imbalance of minerals in blood due to loss of extra salt in sweat leading to dehydration, arrhythmias, fatigue, weakness, heat stroke and rarely death.

## Genetics

The CFTR gene is located at 7q31.2. More than 1900 mutation have been identified of which ‘F508del’ (deletion of three bases coding for phenylalanine at the 508th position) is the most common [12]. Six classes of mutations are described as depicted in Table 1.

**Table 1:** Depicting various classes of mutations, the primary defect and the outcome with examples

Mutation class	Defect	Outcome	Common mutations
I	Protein production	Complete absence of CFTR protein due to premature mRNA termination (nonsense or frame shift mutation) [18, 21, 22]	G542X, W1282X, R553X, 621+G>T
II	Protein processing	Inability of protein to localize to correct cellular location due to abnormal post-translational modifications [18]	F508del, N1303K, A455E
III	Protein regulation	Decreased activity of protein (chloride channel) in response to ATP due to abnormalities of the nuclear binding fold regions [18]	G551D
IV	Protein conduction	Frequency of flow of ions and channel opening duration are reduced though there is generation of chloride currents on stimulation with cAMP [18]	R117H
V	Reduced amount of functional CFTR	Stability of mRNA and/or mature protein is compromised [19, 20]	A455E
VI	Normal amount of functional CFTR	Enhanced turnover due to C-terminus abnormalities	Q1412X

Class I mutations contribute to protein production defect leading to complete absence of CFTR protein, found in 2–5% cases worldwide with the exception of Ashkenazi Jews, in whom 60% of patients carry at least one copy. Class II mutations contribute to protein processing abnormality leading to aberrant localization. It includes F508del which is the most common mutation accounting for 70% of the disease-causing alleles in US. Approximately 50% of the CF patients are homozygous and 90% are heterozygous for this allele. Class III mutations contribute to protein regulation abnormalities leading to a decreased activity. It also includes other mutations especially in regulatory domain. G551D is most common class III mutation. Class IV mutations contribute to protein conduction abnormalities leading to altered frequency of ion flow. Most common mutation is R117H. Class V mutations lead to a reduced amount of functional CFTR protein [13–17] and class VI mutation cause an enhanced protein turnover. Patients carrying Class I–III mutations manifest a more severe form of disease.

However, possible influences of gene modifiers for example TGF-beta1 and mannose-binding lectin have downplayed the clinical significance of a specific combination of mutations [18].

## Complications

Respiratory system complications include Bronchiectasis, Chronic infections leading to pneumonia, growths (nasal polyps), hemoptysis, pneumothorax and eventually respiratory failure.

Digestive system complications include nutritional deficiencies including fat and fat soluble vitamins and diabetes (Nearly 20% of people with cystic fibrosis develop diabetes by age 30). Additionally, progressive hepatic dysfunction, gallstones, intestinal obstruction, intussusception, small intestine bacterial overgrowth (SIBO) and distal intestinal obstruction syndrome (DIOS) may also manifest.

Other complications may include Infertility, Osteoporosis, Electrolyte imbalances and dehydration manifesting as increased heart rate, fatigue, weakness and low blood pressure.

Because of better quality medical interventions and comprehensive care, there is a remarkable increase in percentage of patients (29.2% in 1986 to 49.7% in 2013) surviving above the age of 18 years.

## Treatment

The goals of treatment primarily include:

### Respiratory system

Preventing and controlling lung infections—antibiotics are prescribed. These mainly consist of inhaled forms of azithromycin, tobramycin, aztreonam and levofloxacin. Other antibiotics recommended are ciprofloxacin, cephalexin, amoxicillin and doxycycline depending on the sensitivity patterns [19, 20].

Control of airway inflammation—NSAIDs, inhaled and systemic steroids and cromolyn [21].

Reducing viscoelasticity and removing thick, sticky mucus from the lungs and dilating the airways—inhaled β agonists with humidified oxygen; a 3–6% hypertonic saline solution and dornase alfa are recommended [22–24].

Additionally exercise and physiotherapy including positive expiratory pressure (PEP) device or a high frequency chest wall oscillation device (a percussion vest) is recommended [25].

### GIT

Preventing or treating intestinal blockages—oral rehydration and osmotic laxatives (incomplete blockage) and hyperosmolar contrast enemas (complete DIOS). A balanced electrolyte intestinal lavage solution or enema containing (diatrizoate meglumine and diatrizoate sodium) depending on vomiting status [26]. To prevent recurrence, regular administration of oral polyethylene glycol 3350 may be given for 6 months to 1 year.

Pancreatic insufficiency—pancreatic enzyme replacement therapy (PERT) containing multiple combinations of proteases, lipases and amylases [27].

### Nutrition and electrolyte

Providing appropriate nutrition and preventing dehydration—a high-calorie-fat diet, supplemental vitamins ADEK, and minerals including fluoride and zinc are recommended. Additionally sodium chloride supplementation is given tailored to patient’s age and environmental conditions [28].

Figure 1 summarizes the main abnormalities and treatment approaches in CF patients.

**Fig. 1:** The main pathophysiological dysfunctions and treatment modalities for CF patients. *Inner trapezoid boxes* depict the pathophysiological abnormalities and *outer rectangular boxes* depict the main treatments. The texts connecting the *outer boxes* show non-pharmacological management

In the recent past, Denufosol, an agonist of P2Y2 receptors was tried in CF patients but it eventually failed after early promising results. The detailed analysis is beyond the scope of this review.

## Current and future medicinal products

The current and future therapeutic targets are mainly focused on correcting structural and functional abnormalities of CFTR protein. Additionally, some agents for symptomatic improvement are also in pipeline.

### CFTR modulators

A new group of drugs called CFTR modulators are available which are able to correct the basic defect in CF, i.e. CFTR protein itself though the exact mechanism is not fully elucidated.

#### Ivacaftor

Developed by vertex pharmaceuticals and approved by FDA in 2012 for children ≥6 years having rare mutation, G551D (class III), ivacaftor (Kalydeco) [29] was the first successful medicine to rectify the defective protein and has proven to be very effective in two large multi-centric trials, STRIVE and ENVISION [30, 31]. Marked improvement in FEV^1^, body weight and quality of life were observed. Now FDA has expanded its use in other mutations and also children aged 2–5 years based on the results of KIWI trial [32]. Additionally, a phase IV study (GOAL) also reported improvements in FEV^1^ and FVC, BMI, quality of life and decreased sweat chloride concentration in patients carrying at least one G551D allele. More than 72% patients in this trial also carried F508del as second allele [33]. The G551D mutation causes the channel to act like a locked gate, preventing the trans-conductance of chloride and fluid. The location of channel is proper but the function is impaired. Ivacaftor increases the time of channel in open state. But the main limitation of this therapy is that G551D mutation is present in only 2.3% patients [34]. It is not found to be effective in the most common F508del (class II) mutation because of decreased availability of protein. Additionally, the high cost of therapy may also be a limiting factor (ICER: £335,000–£1,274,000/QALYs gained [35].

#### Lumacaftor

Another CFTR modulator, lumacaftor has shown favorable results in F508del mutation. This is the most common mutation affecting approximately 1/3rd CF population in US and nearly 70% in EU. This mutation affects the heat stability due to misfolding of NBD1 domain and restricts the CFTR in ER for subsequent degradation. It fails to localize to correct epithelial location and achieve normal structure. Increased transport of protein to cell surface was observed in vitro using cultured human bronchial epithelium [36]. Nevertheless, despite increased transport of protein to proper location, no correction of the underlying functional impairment was observed. Moreover, another in vitro study revealed contrasting negative results [37] which were further reinforced by a clinical trial. No significant improvement was observed in FEV^1^, CFQR scores and respiratory exacerbation rates [38].

#### Orkambi

Based on the individual mechanisms, a combination of lumacaftor and ivacaftor (Orkambi) was proposed to correct both, including protein trafficking as well as channel gating abnormalities.

Initially, phase II trials were conducted for both homozygous and heterozygous F508del patients >12 years old but only homozygous patients showed clinically significant results. Two large phase III trials, TRAFFIC and TRANSPORT were conducted with the combination therapy (600 + 250 and 400 + 250 mg versus placebo) in patients ≥12 years with primary endpoint as FEV^1^ improvement at 24 weeks. Patients completing the study were progressed to 48 weeks PROGRESS trial. The isolated as well as pooled results showed a significant improvement in parameters including FEV^1^, reduction of exacerbations, decrease in hospitalizations, increase in BMI and CFQR scores; consistent across different dosage regimens and patient groups. The adverse effects were comparable to placebo group except one case of death during extension phase [39, 40].

Additionally, a phase I study in homozygous children ≤12 years also showed promising results but further advance phase studies are needed [41]. However, when compared to ivacaftor monotherapy in patients having G551D mutation in a separate study, there was significantly less improvement in pulmonary function with combination therapy [42].

Orkambi (lumacaftor + ivacaftor) is approved recently for homozygous F508del patients ≥12 years. Orkambi acts by a two-step method. Lumacaftor assists in moving the defective protein to its correct location and ivacaftor rectifies and enhances its activity eventually increasing the conductance of ions and fluid. Figure 2 shows the possible mechanism of action of Orkambi and other drugs.

**Fig. 2:** Depicting the action of Orkambi (lumacaftor + ivacaftor) and other agents in cystic fibrosis. Orkambi is a combination of two drugs which acts by a two-step method. Lumacaftor assists in moving the defective protein to its correct location and ivacaftor rectifies the gate opening time and enhances its activity eventually increasing the conductance of chloride ions followed by water. Read through agents for example Ataluren increase read through of Premature Termination codon enhancing production of immature protein. Possible “Corrector” drugs act on post translational modifications to increasing stability and reducing degradation by binding to various domains of CFTR. *p-TM* post translational modifications, *GB* golgi bodies, *ER* endoplasmic reticulum

### Possible limitations

Though the arrival of CFTR modulators have improved the CF management but there are still some limitation which include (a) non-significant response in F508del mutation heterozygotes by ivacaftor; (b) need to continue other daily symptomatic treatment; (c) interaction with CYP3A inducers and inhibitors; (d) side effects including elevated transaminases, cataract, oropharyngeal pain and URTI; (e) negligible benefit in <12 years old; (f) need of higher dose up to 600 mg (in case of lumacaftor); and (g) mutual interaction of lumacaftor and ivacaftor leading to increased metabolism of ivacaftor and need of a higher dose combination.

Additionally, because of the multi domain structure and sequential folding of CFTR, no single “corrector drug” can fix all the misfolding in different domains, so a combination of drugs is a must. Moreover, from a clinical trial perspective, there are sample size issues as specific criteria (primary and secondary endpoints) make selection more difficult in already narrowed mutation specific population warranting unique adaptive trial designs.

### Corrector/modifier therapeutic agents in clinical development pipeline

Many other compounds depicting corrector/potentiator activity besides read-through and gene transfer agents and are undergoing various phases of studies as mentioned below.

- *4PBA* (sodium 4-phenylbutarate): though the mechanism of action is not certain but this compound has shown to enhance chloride transport in vitro and in patients having F508del [43].
- *VRT*-*532:* preclinical studies confirmed that this compound corrects the CFTR structural abnormality and increases the protein expression and stability in patients carrying F508del and G551D mutations but showing more affinity for F08del [44, 45].
- *N6022:* increases quantity of CFTR at the epithelium and decrease inflammation. This compound inhibits S-nitrosoglutathione reductase which cause the breakdown of S-nitrosoglutathione, as a result, levels of S-nitrosoglutathione increase which functions as a signaling molecule for protein production [46]. They also limit the binding of HOP (Hsp70/Hsp90 organizing protein) to mature form of CFTR, eventually preventing its degradation. Currently this is in phase 1/2 trials in F508del homozygotes [47].
- *Ataluren (PTC124):* it promotes the read-through of non-sense codons in the mRNA of CFTR (Fig. 1). After promising results in phase II, a phase 3 trial in 2011 also showed a lower rate of decline in lung function. However, another phase 3 trial showed non-significant results (FEV^1^ similar in placebo and drug group) and increased creatinine which was later attributed to inhaled tobramycin [48]. Other trials are currently going on. Additionally a synthetic aminoglycoside NB124 has also depicted a restoration of CFTR activity up to 7% based on the same mechanism of increased PTC suppression [49].
- *Tezacaftor (VX*-*661)* in combination with ivacaftor: a phase 2 trial showed promising results and now this combination is being tried in phase 3. VX-661 is expected to move the defective protein to correct location [50].
- *Riociguat:* though originally approved for treatment of pulmonary hypertension due to its synergistic effect with nitric oxide and stimulation of guanylate cyclase [51], it is currently in phase 2 and preclinical studies have shown positive results regarding expression of CFTR.
- *QBW251:* anticipated as a facilitator/potentiator for channel dynamics, its mechanism is similar to ivacaftor i.e. increasing the channel opening and is expected not to affect the membrane stability of CFTR as by lumacaftor. It is currently undergoing phase 2 [52].
- *N91115(Cavosonstat):* it increases levels of S-nitrosoglutathione which is decreased in CF patients. It has shown to increase the CFTR protein quantity. Just completed phase 1b trial with demonstrated safety and undergoing phase 2a [53].
- *QR*-*010:* it is an antisense oligonucleotide intended to rectify the defective CFTR mRNA. It is given by inhalational route and under phase 1b at present [54].
- Triple therapy of GLPG2665 (corrector) with GLPG2222 (another corrector) and GLPG1837 (potentiator) has shown promising results in early preclinical studies depicting a sixfold more efficacy than Orkambi while early phase human trials are still going on [55–57].
- *CTP656*: it is deuterated ivacaftor which in a phase I trial showed a reduced rate of clearance, increased half-life, significantly improved exposure and better plasma levels [58]. Other corrector drug candidates are FDL160, FDL169 (phase I), FDL392 and FDL304 are also in early developmental pipeline [59].
- *PGM169/GL67A* (plasmid + cationic liposome): is a non-viral CFTR gene transfer agent. It is in phase IIb trial. Repeated nebulization in patients ≥12 years of age showed a modest but significant improvement in lung function but the response is highly varied even FEV^1^ deteriorating in some patients [60]. Additionally, the placebo group received saline based instead of saline based nebulization. Moreover, secondary outcomes like CFTR expression levels, inflammatory markers and NPD showed non-significant results. Another gene transfer agents, Ad5-CB-CFTR, H5.001CBCFTR (with adenovirus) are in phase 1.
- *PTI428*: is projected as a ‘CFTR amplifier’ drug candidate currently in phase I has shown promising results in preclinical studies on HBE cells. Additionally, the PTI-NC-733 is a combination of PTI428 with a corrector and potentiator and has revealed better outcomes in vitro than a combination of ivacaftor and lumacaftor [61, 62].
- *Duramycin (Moli1901/Lancovutide*): activates CaCC in airway epithelium. Has shown improved FEV^1^ in a phase II trial.
- *PDE5 inhibitors*: a study on F508del murine model of CF showed an increased chloride transport in respiratory mucosa on inhalation of PDE5 inhibitors [63]. Also a decrease in sputum neutrophil elastase was found in a clinical study [64]. So, a phase II trial [NCT01132482] is underway to test for the NPD, sweat sodium and chloride concentration, spirometric parameters and lung clearance index. Additionally, the PDE5 inhibitors are also being tested for increased exercise tolerance [NCT02057458].

Cysteamine: by inhibiting transglutaminase 2 (an important multifunctional intermediary in cell autophagy), increases the expression of CFTR and restores its function and decrease inflammatory mediators in murine CF models and epithelial cell lines [65]. A phase II study is done in homo and heterozygous for F508del CF patients in combination with epigallocatechin gallate (which inhibits overactive pleiotropic protein kinase eventually increasing stability of F508del CFTR). The results reported a decrease in sweat chloride concentrations, increased CFTR function, repair of autophagy, decrease in inflammatory cytokines, and improvement in FEV^1^ [66].

Other possible strategy is proteostasis modulation. Growing evidence suggests that CFTR do not works as an isolated ion channel but is a component of wider cellular signaling environment. The functional state of CFTR is modulated by the cellular environment and heterogeneity in cellular signaling. Differences in cellular protein interactomes were found between wild and mutant CFTR, so proteostatis modulation may shift the interactome to a more healthy state thus normalizing the CFTR [67]. As a matter of fact, a deficiency in autophagy pathways as evidenced by reduced autophagosome formation, and the buildup of sequestrosome 1 was discovered in CF airway cells. Myriad proteostasis network interactions have been identified but no human study is done yet. Detailed discussion on these proteostasis networks is beyond the scope of this review.

Another approach is exploration of role of chemical and pharmacological chaperones. They do not act directly on CFTR but on smaller cellular proteins increasing their stability thus modifying the CFTR interactome. Some examples include curcumin and thapsigargin (reducing ER calcium and increasing F508del-CFTR release), Bortezomib (preventing ER associated degradation of F508del-CFTR by increasing HsP70) and Miglustat (inhibitor of α-1,2-glucosidase eventually reducing cytoplasmic degradation of CFTR). Some other compounds include VRT-325, VRT-532 and Corr-4a reducing ubiquitination susceptibility of CFTR. But for most compounds, no corrector activity in humans is yet established. Moreover, there are technical difficulties in bringing these agents to clinical trials and a significant improvement is not anticipated.

Another promising approach is gene editing with the help of nucleases like zinc finger nucleases, transcription activator-like effector nuclease and especially CRISPR/Cas9 (clustered regularly interspaced short palindromic repeats associated with Cas9 nuclease). Engineered nucleases cut the mutant DNA precisely and then wild type DNA is recombined to produce a normal transcript. There is one proof of concept study in intestinal stem cell organoids of CF patients carrying two F508del mutations with CRISPR/Cas9 methodology [68].

In addition, there are many other compounds identified through HTS that may bind and regulate different domains of CFTR and regulate channel activity but these are still in animal experimentation phase.

### Newer therapeutic agents for symptomatic improvement

CF management not only requires CFTR correction and modification but intensive symptomatic treatment targeting inflammation, infection, bronchial hydration and nutrition. Newer drugs targeting these issues are summarized below briefly.

#### Inflammation

*Andecaliximab,* which is an antibody to Matrix metalloproteinase 9 (MMP9) is undergoing phase IIb and expected to reduce inflammation and improve lung function. However, the baseline FEV1 required for this drug is between 40 and 80% limiting its use in very severe CF [69].

Another compound in phase 1 is *POL6014* which is synthesized to block neutrophil elastase function, eventually reducing the tissue destruction and lung inflammation.

*LAU*-*7b* is a fenretinide, a member of retinoid compounds related to vitamin A. Phase 2 study is yet to begin and it is expected to reduce the inflammatory response in CF lungs.

*CTX*-*4430* decreases the production of leukotriene B4, an inflammatory mediator elevated in CF. It is presently undergoing a phase 2 trial [70].

Other anti-inflammatory compounds in clinical development pipeline are *α*-*1 anti*-*trypsin, CTX*-*4430, Elastase Inhibitor AZD9668, JBT*-*101* (phase 2) for reducing inflammation.

#### Hydration and mucus clearance

*AZD5634* is undergoing phase 1b study. It is anticipated to block the sodium channel in CF airway, thus rehydrating and thinning the mucus in the lungs, making it easier to clear.

*SPX*-*101* is another compound designed to block sodium channel function in the lungs, currently undergoing phase II study.

*OrPro (ORP*-*100)* is a modified form of thioredoxin, expected to decrease mucus viscosity in the lungs and improve clearance from the CF airway.

*OligoG* (Alginate Oligosaccharide) has shown to decrease mucus thickness in CF airway. It is currently being tested in phase IIb in Europe and UK. It can be used either as a dry powder or liquid for nebulization [71].

Other agents for rehydration of airway secretions include *bronchitol* currently in phase 3 in US and already approved in UK, Australia and Russia (for patients >18 years); *VX*-*371 (P1037*) presently in phase II for blocking sodium channel and prolonging the duration of hypertonic saline stay [72]; *GSK2225745* acting by silencing ENaC through RNA interference are underway to reach the patients.

#### Nutrition

Liprotamase (Anthera AN-EPI3332) is a pancreatic enzyme replacement for CF-related pancreatic insufficiency undergoing phase 3 study [73].

AquADEKs-2 undergoing phase II is a balanced combination of fat-soluble vitamins and several antioxidants including beta-carotene, mixed tocopherols, coenzyme Q10, mixed carotenoids, and minerals like zinc and selenium.

Oral Glutathione is being tried in phase II as this antioxidant is important for normal lung and GIT function. CF patients have depicted lower glutathione levels and oral glutathione is anticipated to improve growth and decrease gut inflammation [74].

Other agents like enzyme *burlulipase* for pancreatic insufficiency, *lubiprostone* for constipation and *roscovitine* for pulmonary infection are currently being tested at various centers.

## Conclusion

Though there is an improvement in management of CF patients after the approval of CFTR modulators but it is still falling short of mark because in CF, management needs not only the protein rectifiers but also symptomatic treatment and intensive physiotherapy which require concomitant therapies. Myriad genotypes also pose a challenge. Most of the ‘corrector’ drugs in the pipeline are for older children either >12 or 6–12 years of age. Additionally most of these drugs are having serious hepatic and other side effects in addition to high costs. Moreover, many drugs discussed above are still in early clinical phase with limited data and a confirmed beneficial outcome cannot be guaranteed. There is also a need to address the psychological and social burden of disease.

## Future research

Gene engineering techniques and new molecular targets may be explored besides CFTR. Help of modern biology approaches like DNA nanotechnology, systems biology, metabolomics, disease modeling and intracellular protein kinetics may help to unravel new pathways and networks associated with cystic fibrosis and eventually new therapeutic targets. Additionally, the focus should also not be minimized on novel physiotherapy techniques, new drugs for symptomatic improvement and complications prevention.

## References

[1] Reis FJ, Damaceno N (1998). Cystic fibrosis. J Pediatr.

[2] Guggino WB, Banks-Schlegel SP (2004). Macromolecular interaction and ion transport in cystic fibrosis. Am J Respir Crit Care Med.

[3] Johnson LG, Boyles SE, Wilson J, Boucher RC (1995). Normalization of raised sodium absorption and raised calcium-mediated chloride secretion by adenovirus-mediated expression of cystic fibrosis transmembrane conductance regulator in primary human cystic fibrosis airway epithelial cells. J Clin Invest.

[4] Stutts MJ, Canessa CM, Olsen JC (1995). CFTR as a cAMP-dependent regulator of sodium channels. Science.

[5] Cystic fibrosis foundation patient registry: annual data report to the center directors, 2014. https://www.cff.org/2014_CFF_Annual_Data_Report_to_the_Center_Directors.pdf/. Accessed 11 Mar 2016.

[6] Hamosh A, FitzSimmons SC, Macek M, Knowles MR, Rosenstein BJ, Cutting GR (1998). Comparison of the clinical manifestations of cystic fibrosis in black and white patients. J Pediatr.

[7] Cyctic Fibrosis Foundation. About cystic fibrosis. http://www.cff.org/about_cf/what_is_cf. Accessed 17 Mar 2016.

[8] Griese M, Kappler M, Gaggar A, Hartl D (2008). Inhibition of airway proteases in cystic fibrosis lung disease. Eur Respir J.

[9] Davis PB, Davis PB (1993). Pathophysiology of the lung disease in cystic fibrosis. Cystic fibrosis.

[10] Houwen RH, van der Doef HP, Sermet I (2010). Defining DIOS and constipation in cystic fibrosis with a multicentre study on the incidence, characteristics, and treatment of DIOS. J Pediatr Gastroenterol Nutr.

[11] Khoshoo V, Udall JN (1994). Meconium ileus equivalent in children and adults. Am J Gastroenterol.

[12] Orenstein DM, Winnie GB, Altman H (2002). Cystic fibrosis: a 2002 update. J Pediatr.

[13] Moskowitz SM. CFTR-related disorders. http://www.genetests.org. Accessed 27 Oct 2015.

[14] Fanen P, Hasnain A. Cystic fibrosis and the CFTR gene. Atlas of genetic and cytogenetic oncology and hematology, 2001. http://documents.irevues.inist.fr/bitstream/handle/2042/37827/09-2001-CistFibID30032EL.pdf?sequence=3. Accessed 2 Nov 2015.

[15] Antunovic SS, Lukac M, Vujovic D (2013). Longitudinal cystic fibrosis care. Clin Pharmacol Ther.

[16] Abeliovich D, Lavon IP, Lerer I (1992). Screening for five mutations detects 97% of cystic fibrosis (CF) chromosomes and predicts a carrier frequency of 1:29 in the Jewish Ashkenazi population. Am J Hum Genet.

[17] Lukacs GL, Durie PR (2003). Pharmacologic approaches to correcting the basic defect in cystic fibrosis. N Engl J Med.

[18] Mc Kone EF, Emerson SS, Edwards KL, Aitken ML (2003). Effect of genotype on phenotype and mortality in cystic fibrosis: a retrospective cohort study. Lancet.

[19] Moss RB (2002). Long-term benefits of inhaled tobramycin in adolescent patients with cystic fibrosis. Chest.

[20] Konstan MW, Flume PA, Kappler M (2011). Safety, efficacy and convenience of tobramycin inhalation powder in cystic fibrosis patients: the EAGER trial. J Cyst Fibros.

[21] Flume PA, O’Sullivan BP, Robinson KA (2007). Cystic fibrosis pulmonary guidelines: chronic medications for maintenance of lung health. Am J Respir Crit Care Med.

[22] Salvatore D, d’Andria M (2002). Effects of salmeterol on arterial oxyhemoglobin saturations in patients with cystic fibrosis. Pediatr Pulmonol.

[23] Robinson M, Regnis JA, Bailey DL (1996). Effect of hypertonic saline, amiloride, and cough on mucociliary clearance in patients with cystic fibrosis. Am J Respir Crit Care Med.

[24] Quan JM, Tiddens HA, Sy JP (2001). A two-year randomized, placebo-controlled trial of dornase alfa in young patients with cystic fibrosis with mild lung function abnormalities. J Pediatr.

[25] McIlwaine MP, Alarie N, Davidson GF (2013). Long-term multicentre randomised controlled study of high frequency chest wall oscillation versus positive expiratory pressure mask in cystic fibrosis. Thorax.

[26] Colombo C, Ellemunter H, Houwen R (2011). Guidelines for the diagnosis and management of distal intestinal obstruction syndrome in cystic fibrosis patients. J Cyst Fibros.

[27] Stern RC, Eisenberg JD, Wagener JS (2000). A comparison of the efficacy and tolerance of pancrelipase and placebo in the treatment of steatorrhea in cystic fibrosis patients with clinical exocrine pancreatic insufficiency. Am J Gastroenterol.

[28] Borowitz D, Robinson KA (2009). Cystic Fibrosis Foundation evidence-based guidelines for management of infants with cystic fibrosis. J Pediatr.

[29] Kalydeco™ (ivacaftor). Product information. Cambridge: Vertex Pharmaceuticals Inc.; 2012.

[30] Ramsey BW, Davies J, McElvaney NG (2011). A CFTR potentiator in patients with cystic fibrosis and the G551D mutation. N Engl J Med.

[31] Davies JC, Wainwright CE, Canny GJ (2013). Efficacy and safety of ivacaftor in patients aged 6 to 11 years with cystic fibrosis with G551D mutation. Am J Respir Crit Care Med.

[32] Davies JC, Robertson S, Green Y, Rosenfeld M. An open-label study of the safety, pharmacokinetics, and pharmacodynamics of ivacaftor in patients aged 2 to 5 years with CF and CFTR gating mutation: the KIWI study. In: The 28th Annual North American Conference of the Cystic Fibrosis Foundation, Atlanta, GA, October 9–11, 2014.

[33] Rowe SM, Heltshe SL, Gonska T, Donaldson SH, Borowitz D, Gelfond D, Sagel SD, Khan U, Mayer-Hamblett N, Van Dalfsen JM, Joseloff E, Ramsey BW (2014). Network GIotCFFTD. Clinical mechanism of the cystic fibrosis transmembrane conductance regulator potentiator ivacaftor in G551D-mediated cystic fibrosis. Am J Respir Crit Care Med.

[34] http://www.who.int/genomics/publications/en/HGN_WB_04.02_report.pdf. Accessed 27 July 2016.

[35] Whiting P, Al M, Burgers L, Westwood M, Ryder S, Hoogendoorn M, Armstrong N, Allen A, Severens H, Kleijnen J (2014). Ivacaftor for the treatment of patients with cystic fibrosis and the G551D mutation: a systematic review and cost-effectiveness analysis. Health Technol Assess.

[36] Van Goor F, Hadida S, Grootenhuis PD (2011). Correction of the F508del-CFTR protein processing defect in vitro by the investigational drug VX-809. Proc Natl Am Sci USA..

[37] Kopeikin Z, Yukesk Z, Yang H, Bompadre SG (2014). Combined effects of VX-770 and VX-809 on several functional abnormalities on F508del-CFTR channels. J Cyst Fibros.

[38] Clancy JP, Rowe SM, Accurso FJ (2012). Results of a phase IIa study of VX-809, an investigational CFTR corrector compound, in subjects with cystic fibrosis homozygous for the F508del-CFTR mutation. Thorax.

[39] Ramsey B, Boyle MP, Elborn S, et al. Effect of lumacaftor in combination with ivacaftor in patients with cystic fibrosis who are homozygous for F508del-CFTR: pooled results from the phase 3 TRAFFIC and TRANSPORT studies. In: The 28th Annual North American Conference of the Cystic Fibrosis Foundation, Atlanta, GA, October 9–11, 2014.

[40] Wainwright CE, Elborn JS, Ramsey BW, et al. TRAFFIC Study Group; TRANSPORT Study Group. Lumacaftor–ivacaftor in patients with cystic fibrosis homozygous for Phe508del CFTR. N Engl J Med. 2015;373(3):220–31.10.1056/NEJMoa1409547PMC476435325981758

[41] Rosenfeld M, Marigowda G, Liu F, Waltz D. Pharmacokinetics and safety of lumacaftor in combination with ivacaftor in patients aged 6–11 years with CF who are homozygous for F508del-CFTR. In: The 28th annual North American conference of the cystic fibrosis foundation, Atlanta, GA, October 9–11, 2014.

[42] Accurso FJ, Rowe SM, Clancy JP (2010). Effect of VX-770 in persons with cystic fibrosis and the G551D-CFTR mutation. N Engl J Med.

[43] Rubenstein RC, Zeitlin PL (1998). A pilot clinical trial of oral sodium 4-phenylbutyrate (buphenyl) in F508-homozygous cystic fibrosis patients: partial restoration of nasal epithelial CFTR function. Am J Respir Crit Care Med.

[44] Wang Y, Bartlett MC, Loo TW, Clarke DM (2006). Specific rescue of cystic fibrosis transmembrane conductance regulator processing mutants using pharmacological chaperones. Mol Pharmacol.

[45] Wellhauser L, Chiaw PK, Pasyk S (2009). A small-molecule modulator interacts directly with phe508-CFTR to modify its ATPase activity and conformational stability. Mol Pharmacol.

[46] NS30 Pharma. N30 Pharmaceuticals announces first patient treated in clinical trial of N6022 in cystic fibrosis. http://www.n30pharma.com/docs/news/2013-03-12-6022-CF-First-Patient.pdf. Accessed 9 Nov 2015.

[47] National Institutes of Health. Safety and pharmacokinetic study of N6022 in subjects with cystic fibrosis homozygous for the F508del-CFTR mutation (SNO-2) Dec 6, 2012. http://clinicaltrials.gov/show/NCT01746784. Accessed 9 Nov 2015.

[48] Kerem E, Konstan MW, De Boeck K (2014). Ataluren for the treatment of nonsense-mutation cystic fibrosis: a randomised, double-blind, placebo-controlled phase 3 trial. Lancet Respir Med.

[49] Xue X, Mutyam V, Tang L (2014). Synthetic aminoglycosides efficiently suppress cystic fibrosis transmembrane conductance regulator nonsense mutations and are enhanced by ivacaftor. Am J Respir Cell Mol Biol.

[50] A phase 3 study to evaluate the efficacy and safety of ivacaftor and VX-661 in combination with ivacaftor in subjects aged 12 years and older with cystic fibrosis, heterozygous for the F508del-CFTR mutation. https://www.clinicaltrials.gov/ct2/show/NCT02392234?term=vertex+and+661+and+cystic+fibrosis&rank=2. Accessed 7 Jan 2016.

[51] EPAR summary. http://www.ema.europa.eu/docs/en_GB/document_library/EPARSummary_for_the_public/human/002737/WC500165037.pdf. Accessed 7 Jan 2016.

[52] Safety, tolerability, pharmacokinetics, and preliminary pharmacodynamics of QBW251 in healthy subjects and cystic fibrosis patients. https://www.clinicaltrials.gov/ct2/show/NCT02190604?term=QBW251&rank=1. Accessed 12 Jan 2016.

[53] Study of N91115 in patients with cystic fibrosis homozygous F508del-CFTR mutation (SNO4). https://www.clinicaltrials.gov/ct2/show/NCT02275936?term=N91115&rank=2. Accessed 13 Jan 2016.

[54] Dose Escalation Study of QR-010 in Homozygous ΔF508 Cystic Fibrosis Patients. https://clinicaltrials.gov/ct2/show/NCT02532764?term=proqr&rank=1. Accessed 13 Jan 2016.

[55] https://clinicaltrials.gov/ct2/show/record/NCT02662452.

[56] https://clinicaltrials.gov/ct2/show/NCT02707562.

[57] http://www.glpg.com/docs/view/569dedf196364-en.

[58] http://ir.concertpharma.com/releasedetail.cfm?releaseid=935884.

[59] https://clinicaltrials.gov/ct2/show/NCT02359357.

[60] Alton EW, Armstrong DK, Ashby D, Bayfield KJ, Bilton D, Bloomfield EV (2015). Repeated nebulisation of non-viral CFTR gene therapy in patients with cystic fibrosis: a randomised, double-blind, placebo-controlled, phase 2b trial. Lancet Respir Med..

[61] https://clinicaltrials.gov/ct2/show/NCT02718495.

[62] http://www.reuters.com/finance/stocks/companyProfile?symbol=PTI.O.

[63] Lubamba B, Lebacq J, Reychler G (2011). Inhaled phosphodiesterase type 5 inhibitors restore chloride transport in cystic fibrosis mice. Eur Respir J.

[64] Taylor-Cousar JL, Wiley C, Felton LA (2015). Pharmacokinetics and tolerability of oral sildenafil in adults with cystic fibrosis lung disease. J Cyst Fibros.

[65] Luciani A, Villella VR, Esposito S (2012). Targeting autophagy as a novel strategy for facilitating the therapeutic action of potentiators on DeltaF508 cystic fibrosis transmembrane conductance regulator. Autophagy.

[66] Tosco A, De Gregorio F, Esposito S, De Stefano D, Sana I, Ferrari E (2016). A novel treatment of cystic fibrosis acting on-target: cysteamine plus epigallocatechin gallate for the autophagy-dependent rescue of class II-mutated CFTR. Cell Death Diff.

[67] Pankow S, Bamberger C, Calzolari D, Martinez-Bartolomè S, Lavallée-Adam M, Balch WE, Yates JR (2015). ΔF508 CFTR interactome remodelling promotes rescue of cystic fibrosis. Nature.

[68] Schwank G, Koo BK, Sasselli V (2013). Functional repair of CFTR by CRISPR/Cas9 in intestinal stem cell organoids of cystic fibrosis patients. Cell Stem Cell.

[69] A phase 2b, dose-ranging study of the effect of GS-5745 on FEV1 in adult subjects with cystic fibrosis. NCT02759562. https://clinicaltrials.gov/ct2/show/record/NCT02759562. Accessed 15 Mar 2017.

[70] A phase 2, multicenter, randomized, double-blind, placebo-controlled, parallel-group study to evaluate the efficacy, safety, and tolerability of CTX-4430 administered orally once-daily for 48 weeks in adult patients with cystic fibrosis. https://www.clinicaltrials.gov/ct2/show/NCT02443688. Accessed 19 Mar 2017.

[71] A double-blind, randomized, placebo-controlled cross over study of inhaled alginate oligosaccharide (OligoG) administered for 28 days in subjects with cystic fibrosis. https://www.clinicaltrials.gov/ct2/show/NCT02157922. Accessed 21 Mar 2017.

[72] A phase 2a, randomized, double-blind, placebo-controlled, incomplete block, crossover study to evaluate the safety and efficacy of VX-371 in subjects aged 12 years or older with cystic fibrosis, homozygous for the F508del-CFTR mutation, and being treated with Orkambi. https://www.clinicaltrials.gov/ct2/show/NCT02709109.

[73] A phase 3, open-label study evaluating the efficacy and safety of liprotamase in subjects with cystic fibrosis-related exocrine pancreatic insufficiency. https://www.clinicaltrials.gov/ct2/show/NCT02734810. Accessed 15 Mar 2017.

[74] A multi center placebo controlled double blind randomized study evaluating the role of oral glutathione on growth parameters in children with cystic fibrosis. https://clinicaltrials.gov/ct2/show/NCT03020719. Accessed 13 Mar 2017.

